This article has been retracted.

# *Qibin Tongbian* Decoction in the Treatment of Diabetic Constipation and Its Influence on the Intestinal Environment and the Incidence of Adverse Reactions: A Randomized Trial

**DOI:** 10.1155/2022/5373765

**Published:** 2022-04-30

**Authors:** Cunxiang Tang, Wenyuan Pu, Zhaowei Shan

**Affiliations:** Nanjing University of Chinese Medicine, Nanjing, China

## Abstract

**Objective:**

This study aimed to study the clinical efficacy of *Qibin Tongbian* decoction in the treatment of diabetic constipation and its influence on the intestinal environment and the incidence of adverse reactions.

**Methods:**

In this prospective study, a total of 62 patients with diabetic constipation admitted to our hospital from June 2020 to March 2021 were recruited and assigned at a ratio of 1 : 1 to receive either traditional treatment (control group) or *Qibin Tongbian* decoction (experimental group). Outcome measures included clinical efficacy, intestinal environment, and incidence of adverse reactions.

**Results:**

Qibin Tongbian decoction was associated with significantly higher efficacy and a lower TCM symptom score versus conventional treatment (*P* < 0.05). *Qibin Tongbian* decoction resulted in significantly lower fasting plasma glucose (FPG) levels and 2-hour postprandial plasma glucose (2hPG) levels versus conventional treatment (*P* < 0.05). Patients receiving *Qibin Tongbian* decoction showed significantly lower constipation symptom scores and PAC-QOL scores versus conventional treatment (*P* < 0.05). *Qibin Tongbian* decoction resulted in a significantly larger number of bifidobacteria and enterococci and a smaller number of yeasts versus conventional treatment (*P* < 0.05). *Qibin Tongbian* decoction was associated with a significantly lower incidence of adverse reactions and recurrence rate versus conventional treatment (*P* < 0.05).

**Conclusion:**

*Qibin Tongbian* decoction combined with conventional TCM therapy yields a promising effect in the treatment of diabetic constipation. It can improve the intestinal environment of patients, mitigate the symptoms of constipation, enhance the quality of life of patients, and reduce the incidence of adverse reactions, so it is worthy of promotion and application.

## 1. Introduction

As a common clinical symptom of diabetic autonomic neuropathy involving the digestive system, diabetic constipation is associated with the damage of intestinal mucosal epithelial cells caused by increased blood sugar, decreased sensitivity of the large intestine, and autonomic neuropathy of the large intestine [1, 2]. Excessive blood sugar can result in fluid deficiency in the body, causing dry stools and difficulty in defecation. Therefore, maintenance of a proper diet is crucial for diabetic patients; for example, the intake of plant fiber foods can promote intestinal peristalsis and also facilitate the propagation of intestinal probiotic flora [2, 3]. Constipation may aggravate the patient's psychological burden and negative emotions, which in turn increase the secretion of insulin-antagonistic hormones and lead to blood sugar instability [3, 4]. The current treatment focuses on blood sugar control. According to the patient's symptoms, the use of drugs that promote gastrointestinal motility can increase bowel movement and defecation frequency, thereby alleviating the symptoms of constipation. Discouragingly, the symptoms of constipation would reoccur after drug withdrawal, emanating a somber effect [5–7]. Previous studies have shown that TCM emphasizes dialectical treatment and produces satisfying results in the treatment of diabetic constipation [7, 8]. Common symptoms of constipation include abdominal pain, bloating, loss of appetite, nervousness, and insomnia, which may lead to the formation of hemorrhoids, bleeding anal fissures, and perianal infections. Since the elderly are often combined with hypertension, chronic bronchitis, acute and chronic cardiovascular and cerebrovascular pathologies, cataracts, glaucoma, and severe constipation, elderly patients are prone to defecation difficulties, and excessive straining of the bowels may induce cerebrovascular rupture, heart failure, cardiac arrest, colon rupture perforation, and blindness, which seriously compromises the quality of life of elderly diabetic patients and even causes serious harm. Therefore, this study attempts to explore the clinical efficacy of *Qibin Tongbian* decoction combined with conventional TCM treatment of diabetic constipation, and its influence on the intestinal environment and the incidence of adverse reactions in patients.

## 2. Materials and Methods

### 2.1. 1Subjects

In this prospective study, a total of 62 patients with diabetic constipation admitted to our hospital from June 2020 to March 2021 were recruited and assigned (1 : 1) to a control group or an experimental group. The control group consisted of 13 males and 18 females, aged 48–69 (55.44 ± 12.30) years; the course of diabetes was 4–10 (6.52 ± 3.81) years; and constipation course was 1–4 (2.61 ± 1.56) years. The experimental group consisted of 15 males and 16 females, aged 45–70 (56.53 ± 11.96) years; the course of diabetes was 3–9 (5.87 ± 3.74) years; and constipation course was 2–5 (3.22 ± 1.69) years. The two groups showed similar baseline data (*P* > 0.05). The study was approved by the Ethics Committee of Nanjing University of Chinese Medicine with ethics certificate number 2019-12-11, and all patients and families gave their informed consent.

### 2.2. Inclusion Criteria and Exclusion Criteria

Inclusion criteria are as follows: ① all patients met the relevant diagnostic criteria of diabetes and Rome III functional constipation; ② all patients met the relevant diagnostic criteria of Qi-Yin deficiency and intestine dryness in TCM; ③ aged 18∼75 years; ④ with a diabetic history of more than 3 years and chronic constipation of more than 6 months; ⑤ fasting blood glucose was controlled below 7 mmol/L, 2 hours after-meal blood glucose was controlled below 10 mmol/L, and HbA1c was controlled below 7.0%; ⑥ no laxatives such as magnesium sulfate and lactulose, no anthraquinones, and gastrointestinal motility drugs were used in the first week before the experiment; ⑦ no specific treatment has been taken in the past month; and ⑧ the patients and their families knew the purpose and process of this study and signed an informed consent form.

Exclusion criteria are as follows: ① those who did not meet diagnostic criteria; ② pregnant or breastfeeding women; ③ with diabetic ketosis, ketoacidosis, or severe infection in the last half month; ④ with severe intestinal organic lesions or constipation caused by drug-derived factors; ⑤ with serious diseases of the cardiopulmonary, brain, liver, and kidney systems; ⑥ with serious mental or psychological diseases; and ⑦ patients participating in clinical trials of other drugs.

## 3. Methods

Patients in both groups received basic treatment for diabetes in the endocrine department, including hypoglycemic drugs, dietary conditioning, exercise therapy, and psychological therapy, to maintain the stability of blood glucose.

The control group received oral mosapride citrate dispersible tablet (Xinluona, Chengdu Kanghong Pharmaceutical Group Co., Ltd), 5 mg each time, 3 times a day, for 2 weeks. The experimental group received *Qibin Tongbian* decoction. Composition of the prescription: Astragalus 15 g, Atractylodes 10 g, hemp seed 10 g, Immaturus aurantii 10 g, peach kernel 10 g, cistanche 10 g, Trichosanthis seed 10 g, areca nut 10 g, Humifuse euphorbia herb 10 g, Cortex lycii radicis 10 g, and Radix ophiopogonis 15 g. The herbs were decocted in water and filtered to obtain the decoction, 1 dose per day with half dose taken in the morning and a half in the evening, for a course of 4 weeks.

### 3.1. Observation Indicators and Evaluation Criteria

(1) TCM symptom score and clinical efficacy: the TCM symptom score of the two groups of patients was assessed with reference to the *Guiding Principles for Clinical Research of New Chinese Medicines* [9]. The clinical efficacy was evaluated by the defecation frequency. Cured: the bowel movement frequency is more than 5 times per week and the bowel movement is smooth after treatment, and the stools are loose; markedly effective: the defection frequency is 3–4 times per week and the bowel movement is smooth, and the stool is loose or the bowel movement frequency is more than 5 times per week; effective: the bowel movement frequency is 3–5 times per week, and the bowel movement is smooth, but the stool is dry; and ineffective: the clinical symptoms have not changed or the defection frequency is less than 3 times per week. The total efficacy = (cured + markedly effective + effective)/total number of cases × 100%. (2) The fasting plasma glucose (FPG) and 2-hour postprandial plasma glucose (2hPG) of patients before and after treatment were recorded and compared. (3) Symptoms of constipation: symptoms of constipation including the frequency of defecation, the degree of difficulty in defecation, the feeling of incomplete defecation, duration of defection, abdominal pain, defecation assistance methods, and the number of attempts of unsuccessful defecation per day were evaluated using the Cleveland scale. The full score is 26 points, and a higher score suggests more severe constipation symptoms. (4) Quality of life: the quality of life of patients with constipation was scored by Patient Assessment of Constipation Quality of Life (PAC-QOL), which was scored from the four dimensions of physiology, psychology, worry, and satisfaction, with 28 items. 0 points represent none, a score of 1 point represents a slight condition, a score of 2 points represents a general condition, a score of 3 points represents a serious condition, and a score of 4 points represents a very serious condition. The scores of the 28 items of the patient were recorded. The higher the score, the lower the quality of life of the patient. (5) Before and after treatment, a sufficient amount of feces was obtained and placed in a clean stool box to detect the contents of bifidobacteria, enterococci, and yeasts in the patient's body using real-time polymerase chain reaction (PCR). (6) The incidence of adverse reactions was compared between the two groups of patients, including nausea, vomiting, and abdominal pain. (7) The patients were followed up for 6 months to compare the recurrence of constipation between the two groups.

### 3.2. Statistical Analysis

The data were statistically analyzed by SPSS 20.0, and GraphPad Prism 7 (GraphPad Software, San Diego, USA) was used to plot graphics. The count data were tested by the chi-square test and expressed as (*n*(%)), and measurement data were examined by *t*-test and expressed as (*x* ± *s*). Differences were considered statistically significant at a *P* value of <0.05.

## 4. Results

### 4.1. TCM Symptom Score and Clinical Efficacy

Before treatment, the TCM symptom scores were comparable between the two groups (*P* > 0.05). *Qibin Tongbian* decoction was associated with a significantly higher efficacy (96.67% vs. 83.33%) and a lower TCM symptom score versus conventional treatment (*P* < 0.05). See Tables 1 and 2.

### 4.2. FPG and 2hPG Levels

Before treatment, the FPG and 2hPG levels of the two groups of patients were not statistically different (*P* > 0.05). *Qibin Tongbian* decoction resulted in significantly lower FPG and 2hPG levels versus conventional treatment (*P* < 0.05). See Figures 1(a) and 1(b).

### 4.3. Constipation Symptom Scores and PAC-QOL Scores

Before treatment, no statistical difference in the scores of constipation symptoms and PAC-QOL scores was observed between the two groups (*P* > 0.05). Patients receiving *Qibin Tongbian* decoction showed significantly lower constipation symptom scores and PAC-QOL scores versus conventional treatment (*P* < 0.05). See Figures 2(a) and 2(b).

### 4.4. Changes in Intestinal Flora

The two groups showed no significant differences in terms of the number of bifidobacteria, enterococci, and yeasts before treatment (*P* > 0.05). *Qibin Tongbian* decoction resulted in a significantly larger number of bifidobacteria and enterococci and a smaller number of yeasts versus conventional treatment (*P* < 0.05). See Table 3.

### 4.5. Incidence of Adverse Reactions

*Qibin Tongbian* decoction was associated with a significantly lower incidence of adverse reactions (1.67%) versus conventional treatment (11.67%) (*P* < 0.05). See Table 4.

### 4.6. Recurrence of Constipation

There were 50 patients with effective treatment in the control group and 58 patients in the experimental group. The patients given *Qibin Tongbian* decoction showed a significantly lower recurrence rate versus conventional treatment (*P* < 0.05). See Table 5.

## 5. Discussion

Diabetic constipation is caused by multiple factors, such as decreased gastrointestinal motility caused by autonomic nerve dysfunction consequent to diabetes, gastrointestinal hormone secretion disorders resulting from prolonged hyperglycemia, and imbalanced intestinal flora [10, 11]. In traditional Chinese medicine, the large intestine is the organ of conduction to discharge stools from the body. Long-term unhealthy eating habits may generate internal heat, cause an imbalance of spleen and stomach function, and result in the obstruction of damp heat and turbidity in the intestinal tract and the difficulty in discharging stools [11, 12]. TCM acupuncture therapy is to stimulate the function of enteric nerve cells through acupuncture points, which can increase the nerve excitability of the patient, enhance the muscle strength of the pelvic floor muscle, and alleviate the symptoms of constipation caused by pelvic floor muscle relaxation [13, 14]. Abdominal acupoint massage can increase the tension of the muscles of the gastrointestinal lining and the function of the lymphatic system, activate the secretion of the gastrointestinal organs, boost gastrointestinal peristalsis, promote digestion, absorption, and excretion of food, and resolve constipation [15, 16]. The Astragalus and Codonopsis in *Qibin Tongbian* decoction can nourish the lung and spleen; angelica, hemp seed, white honey, and cistanche play a role in nourishing blood, moistening the intestines, and relaxing the bowels; tangerine peel exerts the effects of regulating *Qi*, promoting spleen, drying dampness, and reducing phlegm; white Atractylodes rhizome and Fructus aurantii have the effect of invigorating the spleen and regulating *Qi*; betel nut slices yield a satisfying result in regulating *Qi* and dredging stagnation, unblocking the accumulation; peach kernels function well in promoting blood circulation, removing blood stasis, and moisturizing the intestines; fried raspberry seeds have the property of treating constipation; and licorice can reconcile the above medicines [9, 17, 18].

In this study, *Qibin Tongbian* decoction was associated with a significantly higher efficacy (96.67% vs. 83.33%) and lower FPG and 2hPG levels versus conventional treatment, indicating that *Qibin Tongbian* decoction produces a favorable effect on diabetic constipation. Remarkably, patients receiving *Qibin Tongbian* decoction showed significantly lower constipation symptom scores and PAC-QOL scores versus conventional treatment, which was consistent with the research results of Li et al. [19], suggesting that *Qibin Tongbian* decoction can mitigate the symptoms of constipation and improve the quality of life of patients. Additionally, *Qibin Tongbian* decoction resulted in a significantly larger number of bifidobacteria and enterococci and a smaller number of yeasts versus conventional treatment, indicating that *Qibin Tongbian* decoction can improve the intestinal environment of patients with constipation and boost the function of intestinal peristalsis. Furthermore, the incidence of adverse reactions in the experimental group was 1.67% and that in the control group was 11.67%, indicating that *Qibin Tongbian* decoction for diabetic constipation can reduce adverse reactions. Encouragingly, the patients with robust effects were followed up for 6 months, and the results showed that the recurrence rate of patients in the control group was higher than the experimental group (26% vs 6.90%), and the results of this study are in line with a previous study [20] stating that *Qibin Tongbian* decoction can notably reduce the recurrence rate of the experimental group in contrast with the control group (16.59% vs 44.15%). The above results suggest a promising effect of *Qibin Tongbian* decoction in treating diabetic constipation and reducing the recurrence rate of constipation. Qibin Tongbian decoction is mostly used to nourish the kidney and strengthen the spleen. Constipation is closely related to the kidney. A deficiency in kidney Yin results in a loss of intestinal moistening and dryness, while a deficiency in kidney Yang results in an inability to warm and moisten the intestines. The spleen and stomach are the sources of Qi and blood, with the main function of transformation of nutrients, so spleen Qi deficiency will reduce the function of nutrient intake. The lung and large intestines are closely associated. Lung Qi deficiency leads to weakness of large intestine conduction, and blood deficiency prevents fluid from nourishing the large intestine; Yin deficiency of the lung results in dryness of the large intestine and loss of intestinal moistening, both of which can lead to dry stools and difficult discharge, resulting in constipation. Due to prolonged dryness, liver depression, and Qi stagnation, blood stasis blocks the ligaments, and fluid cannot penetrate the large intestine, resulting in fluid deficiency and intestinal dryness, which can aggravate the condition.

Qirong Runchang oral solution is effective in the treatment of diabetic constipation in the elderly, especially in elderly diabetic patients with deficiency of Qi and Yin, deficiency of spleen and kidney, and loss of bowel moistening as identified by traditional Chinese medicine, with a fast onset of action and a significant laxative effect. Its short-term use can significantly improve the patient's bowel movement and relieve constipation symptoms, and long-term use can ameliorate the symptoms of general body weakness, thus enhancing the patient's quality of life significantly. The drug features gentle action, long maintenance, no significant effect on glycemic control in elderly diabetic patients, and no significant adverse drug reactions, which is worthy of clinical reference and use.

The innovation of this study is the use of Qibin Tongbian decoction in combination with conventional Chinese medicine for the treatment of diabetic constipation. The limitation of this study is the absence of long-term extensive follow-up data to determine the long-term efficacy of diabetic patients, which requires additional follow-up time in the future to obtain more clinical information.

## 6. Conclusion

A combination of *Qibin Tongbian* decoction is a preferred option for diabetic constipation. It can improve the patient's intestinal environment and patient's constipation symptoms, upgrade the patient's quality of life, and reduce the incidence of adverse reactions, with a high safety profile.

## Figures and Tables

**Figure 1:** Comparison of the FPG levels and 2hPG levels. Note: (a). The abscissa indicates before and after treatment, and the ordinate indicates the FPG level, mmol/L; the FPG levels of children in the control group before and after treatment were 9.36 ± 0.25 mmol/L and 7.06 ± 0.18 mmol/L, respectively; the FPg levels of children in the experimental group before and after treatment were 9.41 ± 0.19 mmol/L and 6.05 ± 0.23 mmol/L, respectively; *∗* indicates that there is a significant difference in FPG levels before and after treatment in the control group (*P* < 0.05); *∗∗* indicates that there is a significant difference in FPG levels before and after treatment in the experimental group (*P* < 0.01); *∗∗∗* indicates that there is a significant difference in FPG levels between the experimental group and the control group after treatment (*P* < 0.001). (b). The abscissa indicates before and after treatment, and the ordinate indicates the level of 2hPG, mmol/L; the 2hPG levels of children in the control group before and after treatment were 13.59 ± 0.43 mmol/L and 11.14 ± 0.52 mmol/L, respectively; the 2hPG levels of children in the experimental group before and after treatment were 13.67 ± 0.54 mmol/L and 9.03 ± 0.55 mmol/L, respectively; *∗* indicates that there is a significant difference in 2hPG levels before and after treatment in the control group (*P* < 0.05); *∗∗* indicates that there is a significant difference in 2hPG levels before and after treatment in the experimental group (*P* < 0.01); *∗∗∗* indicates that there is a significant difference in 2hPG levels between the experimental group and the control group after treatment (*P* < 0.001).

**Figure 2:** Comparison of constipation symptom scores and PAC-QOL scores. Note: (a). The abscissa indicates before and after treatment, and the ordinate indicates the score of constipation symptoms, points; the scores of constipation symptoms before and after treatment in the control group were 19.80 ± 2.03 points and 13.56 ± 1.47 points, respectively; the scores of constipation symptoms before and after treatment in the experimental group were 19.76 ± 3.01 points and 7.6 ± 1.38 points, respectively; *∗* indicates that there is a significant difference in the scores of constipation symptoms in the control group before and after treatment (*P* < 0.05); *∗∗* indicates that there is a significant difference in the scores of constipation symptoms in the experimental group before and after treatment ( *P* < 0.01); *∗∗∗* indicates that there is a significant difference in the scores of constipation symptoms between the experimental group and the control group after treatment (*P* < 0.001). (b). The abscissa represents before and after treatment, and the ordinate represents PAC-QOL score, points; the PAC-QOL scores of children in the control group before and after treatment were 76.44 ± 4.25 points and 49.61 ± 4.30 points, respectively; the PAC-QOL scores of the children in the experimental group were 77.06 ± 5.12 and 38.57 ± 7.41 points before and after treatment, respectively; *∗* indicates that the PAC-QOL scores of children in the control group were significantly different before and after treatment (*P* < 0.05); *∗∗* indicates that the PAC-QOL scores of children in the experimental group were significantly different before and after treatment (*P* < 0.01); *∗∗∗* indicates that there is a significant difference in the scores of constipation symptoms between the experimental group and the control group after treatment (*P* < 0.001).

**Table 1:** TCM symptom complex score and clinical efficacy.

	*n*	TCM score	
		Before	After

Control group	31	33.29 ± 9.25	18.28 ± 6.57
Experimental group	31	35.95 ± 7.58	12.05 ± 5.25
*T*		1.238	4.125
*P*		0.220	<0.001

**Table 2:** Clinical efficacy of the two groups (*n*(%)).

	*n*	Cured	Markedly effective	Effective	Ineffective	Total efficacy

Control group	31	4	6	10	11	20
Experimental group	31	9	7	12	3	28
*X* ^2^						5.905
*P*						0.015

**Table 3:** Comparison of changes in intestinal flora ($\bar{x}$ ± *s*).

	*n*	Bifidobacterium		Enterococcus		Yeast	
		Before	After	Before	After	Before	After

Control group	31	7.45 ± 1.69	8.14 ± 1.02	7.91 ± 1.26	8.48 ± 1.12	4.49 ± 0.68	3.95 ± 0.58
Experimental group	31	7.46 ± 1.82	9.65 ± 1.13	7.85 ± 1.29	9.37 ± 1.40	4.57 ± 0.76	3.04 ± 0.23
*t*		0.022	5.523	0.185	2.764	0.437	8.120
*P*		0.982	<0.001	0.853	0.008	0.664	<0.001

**Table 4:** Comparison of the incidence of adverse reactions (*n*(%)).

	*n*	Vomiting	Nausea	Abdominal pain	Total incidence

Control group	31	3	2	4	9
Experimental group	31	0	0	1	1
*X* ^2^					7.631
*P*					0.006

**Table 5:** Comparison of the recurrence of constipation (*n*(%)).

Group	Recurrence	Non-recurrence

Control group	12 (38.71)	19 (61.29)
Experimental group	3 (9.68)	28 (90.32)
*X* ^2^	7.123	
*P*	0.008	

## Data Availability

The data used to support the findings of this study are available from the corresponding author upon request.
